The article "Consumption of pomegranates improves synaptic function in a transgenic mice model of Alzheimer's disease" was retracted in 2025. Reasons: duplicated images; original data or images not available; concerns about the images; concerns about the authorship.

# Consumption of pomegranates improves synaptic function in a transgenic mice model of Alzheimer's disease

**DOI:** 10.18632/oncotarget.10905

**Published:** 2016-07-28

**Authors:** Nady Braidy, Musthafa Mohamed Essa, Anne Poljak, Subash Selvaraju, Samir Al-Adawi, Thamilarasan Manivasagm, Arokiasamy Justin Thenmozhi, Lezanne Ooi, Perminder Sachdev, Gilles J. Guillemin

**Affiliations:** ^1^ Centre for Healthy Brain Ageing, School of Psychiatry, Faculty of Medicine, University of New South Wales, Sydney, Australia; ^2^ Department of Food Science and Nutrition, College of Agricultural and Marine Sciences, Sultan Qaboos University, Al Khoudh, Oman; ^3^ Ageing and Dementia Research Group, Sultan Qaboos University, Al Khoudh, Oman; ^4^ College of Medicine and Health Sciences, Sultan Qaboos University, Al Khoudh, Oman; ^5^ Department of Biochemistry and Biotechnology, Annamalai University, Tamil Nadu, India; ^6^ Illawarra Health and Medical Research Institute, University of Wollongong, NSW, Australia; ^7^ Neuropsychiatric Institute, The Prince of Wales Hospital, Sydney, Australia; ^8^ Neuroinflammation Group, MND and Neurodegenerative Diseases Research Centre, Macquarie University, NSW, Australia

**Keywords:** pomegranates, synapse, inflammation, amyloid beta protein, amyloid precursor protein, Gerotarget

## Abstract

Alzheimer's Disease (AD) is a progressive neurodegenerative disorder characterized by extracellular plaques containing abnormal Amyloid Beta (Aβ) aggregates, intracellular neurofibrillary tangles containing hyperphosphorylated tau protein, microglia-dominated neuroinflammation, and impairments in synaptic plasticity underlying cognitive deficits. Therapeutic strategies for the treatment of AD are currently limited. In this study, we investigated the effects of dietary supplementation of 4% pomegranate extract to a standard chow diet on neuroinflammation, and synaptic plasticity in APPsw/Tg2576 mice brain. Treatment with a custom mixed diet (pellets) containing 4% pomegranate for 15 months ameliorated the loss of synaptic structure proteins, namely PSD-95, Munc18-1, and SNAP25, synaptophysin, phosphorylation of Calcium/Calmodulin Dependent Protein Kinase IIα (p-CaMKIIα/ CaMKIIα), and phosphorylation of Cyclic AMP-Response Element Binding Protein (pCREB/CREB), inhibited neuroinflammatory activity, and enhanced autophagy, and activation of the phophoinositide-3-kinase-Akt-mammalian target of rapamycin signaling pathway. These neuroprotective effects were associated with reduced β-site cleavage of Amyloid Precursor Protein in APPsw/Tg2576 mice. Therefore, long-term supplementation with pomegranates can attenuate AD pathology by reducing inflammation, and altering APP-dependent processes.

The article "Consumption of pomegranates improves synaptic function in a transgenic mice model of Alzheimer's disease" was retracted in 2025. Reasons: duplicated images; original data or images not available; concerns about the images; concerns about the authorship.

## INTRODUCTION

Alzheimer's Disease (AD) is a progressive neurodegenerative disorder characterized clinically by progressive cognitive and memory impairments [1]. Recent epidemiological studies have shown that at least 36.5 million individuals are affected by AD worldwide, with new AD diagnosis reported every 7 seconds [2]. Ageing represents the main risk factor for AD and its prevalence is expected to increase exponentially with age [1, 3-5]. The aetiology and exact neuropathogenesis of AD remain unclear. However, AD is thought to be a complex multi-factorial disorder, and no effective therapeutic agent is available to slow down or prevent disease progression [6, 7].

The main pathological hallmarks of AD is the formation of extracellular Amyloid-Beta (Aβ) deposits called senile plaques, and twisted intracellular neurofibrillary tangles containing hyperphosphorylated tau, a microtubular protein [8]. Aβ plaques can induce synaptic loss in the neocortex and limbic system, leading to neuronal injury. Aβ can also induce neuronal damage through activation of microglia, the resident immunoregulatory cells in the brain, leading to the production and release of neurotoxic and pro-inflammatory cytokines, such as Tumor Necrosis Factor (TNF)-α, Interleukin (IL)-1β, and highly volatile free radicals [9]. Microglial activation represents a critical process to facilitate the clearance of Aβ from the brain *via* endocytosis [10, 11]. Therefore, therapeutic strategies targeting neuroinflammation and microglial activation are highly desirable [12-15].

The generation of Aβ is dependent on the proteolytic processing of Amyloid Precursor Protein [16] by α-secretase, β-secretase (BACE1), and γ-secretase. α-secretase is responsible for the cleavage of APP at the luminal region, thus preventing the formation of neurotoxic Aβ aggregates and plaques [17, 18]. BACE1 is responsible for the cleavage of full length APP on the N-terminus of Aβ, consequently leading to the formation of smaller soluble ectodomain fragment (sAPP-β), and a larger C-terminal fragment (C99) [19-22]. γ-secretase catalyses the formation of Aβ from the C99 fragment [23]. Given the significance of Aβ in AD pathology, therapeutic strategies aimed at interfering with the processing of APP are warranted.

Synaptic dysfunction represents another pathological presentation of AD. Synaptic plasticity is crucial for the maintenance of optimal memory and learning [24-26]. Since impairments in synaptic plasticity precede synaptic loss, changes to synaptic regulatory protein may represent an important biomarker for disease progression and cognitive impairments [27, 28]. An important example is Mammalian Target Of Rapamycin (mTOR), a kinase associated with the maintenance of synaptic plasticity by modulating the anabolism of protein [29].

The article "Consumption of pomegranates improves synaptic function in a transgenic mice model of Alzheimer's disease" was retracted in 2025. Reasons: duplicated images; original data or images not available; concerns about the images; concerns about the authorship.

Pomegranates (*Punica granatum Linn*.) are composed of high concentrations of polyphenols compared to other fruits and vegetables [30-43]. Pomegranates have been extensively used for the treatment of several degenerative diseases in Unani, Ayurvedic and Chinese systems of medicine [44]. Dietary supplementation of pomegranate juice attenuated neurodegeneration in neonatal mice subjected to maternal hypoxic-ischemic brain injury [45, 46]. We and others have previously shown that pomegranate supplementation with diet significantly reduced oxidative stress in brain [47-49]. This effect of pomegranate was likely through inhibition of Aβ accumulation, which in turn significantly attenuated oxidation of lipid and protein, restored Acetylcholinesterase (AChE) activity, maintained endogenous antioxidant capacity at near physiological levels in brain tissues of APPsw/Tg2576 mice, and improved spatial learning deficits [47-49].

The Tg2576 mice express APP KM670/671NL Swedish mutation, and demonstrates progressive age-dependent behavioural deficits associated with increased Aβ deposition. Moreover, this transgenic mice model exhibit decreased motor coordination, increased learning and memory deficits, and elevations in oxidative stress markers. Previous studies have identified significant memory impairment, and hippocampal neurodegeneration in Tg2576 mice. The current study explores the effect of pomegranate supplementation on stress in the brain, synaptic plasticity, neuroinflammation, and Aβ production in the AD transgenic mice, and examines potential disease-related modifications to the expression of synaptic plasticity-related proteins, activation of the PI3K/Akt/mTOR pathway, neuroinflammation, and altered amyloidogenic processing.

## RESULTS

### Long-term supplementation with 4% pomegranates improved synaptic structure protein in APPsw/Tg 2576

Numerous studies have shown that the expression of synaptic structural protein is reduced in the brains of AD mice compared to wild-type controls [50, 51]. We have shown that the protein expression of PSD-95, Munc18-1, SNAP25, synaptophysin, p-CaMKIIα/ CaMKIIα, and pCREB/CREB were significantly increased (*p* < 0.05) in the brain in APPsw/Tg 2576 receiving a diet supplemented with 4% pomegranates for 15 months than in APPsw/Tg 2576 mice receiving a standard chow diet (Figure 1).

**Figure 1:** Synaptic structural proteins in brain homogenates detected by Western blot analysis The levels of PSD-95, Munc18-1, SNAP25, synaptophysin, p-CaMKIIα/ CaMKIIα, and pCREB/CREB in the brains of mice fed 4% pomegranate diet for 15 months. Treatment I: Wild type (non-transgenic) control of the APPsw mice fed with regular diet; Treatment II: APPsw mice also fed with regular diet; and Treatment III: APPsw mice fed with 4% pomegranate fruit diet. **A.** The blot shown is representative tracings of an experiment done six times. **B.** Graphs are mean ± S.E brains from tissue obtained from six rodents for each treatment group. Each bar of the quantification graph represents the corresponding band for each age group. Significance ^*^p < 0.01 compared to wild-type mice fed with regular diet, ^#^*p* < 0.01 compared to APPsw transgenic mice fed with regular diet.

The article "Consumption of pomegranates improves synaptic function in a transgenic mice model of Alzheimer's disease" was retracted in 2025. Reasons: duplicated images; original data or images not available; concerns about the images; concerns about the authorship.

We also assessed the mRNA expression of genes encoding for two important neurotrophic factors, BDNF and IGF-1 (Figure 2). Our data shows that both BDNF and IGF-1 are significantly increased in the brain by 15 months of treatment with a 4% pomegranate diet compared to APPsw/Tg 2576 mice receiving a standard chow diet.

**Figure 2:** mRNA expression of genes encoding for neurotrophic factors and proinflammatory markers Treatment I: Wild type (non-transgenic) control of the APPsw mice fed with regular diet; Treatment II: APPsw mice also fed with regular diet; and Treatment III: APPsw mice fed with 4% pomegranate fruit diet. The levels of two important neurotrophic factors, BDNF and IGF-1, and the proinflammatory cytokines, tnf-α, il-1β, iNOS, ccl2, and il-10, in the brains of mice fed 4% pomegranate diet for 15 months were determined using real-time polymerase chain reactions. Graphs are mean ± S.E brains from tissue obtained from six rodents for each treatment group. Significance ^*^p < 0.01 compared to wild-type mice fed with regular diet, ^#^*p* < 0.01 compared to APPsw transgenic mice fed with regular diet.

### Long-term supplementation with 4% pomegranates reduces neuroinflammation in APPsw/Tg 2576

It is well established that neuroinflammation plays a pivotal role in the pathogenesis of AD [12-15]. We examined whether long-term treatment with 4% pomegranates attenuated neuroinflammatory activity in APPsw/Tg 2576. To determine this, we quantified the expression of inflammatory genes in the brain. Our data shows that the expression of tnf-α, il-1β, iNOS, ccl2, and il-10 were significantly decreased by diet supplemented with 4% pomegranates for 15 months (*p* < 0.05) (Figure 2).

### Autophagy is enhanced by long-term supplementation with 4% pomegranates in APPsw/Tg 2576

Apart from the improvements in synaptic protein expression and inhibition of neuroinflammation, we assessed the effects of 4% pomegranate supplementation on autophagy. We observed that dietary supplementation with 4% pomegranates significantly induced autophagy, as shown by increased protein expression of Beclin-1 (bcl1) and Lipidated LC-3 (LC-3 type II) (*p* < 0.05) (Figure 3).

The article "Consumption of pomegranates improves synaptic function in a transgenic mice model of Alzheimer's disease" was retracted in 2025. Reasons: duplicated images; original data or images not available; concerns about the images; concerns about the authorship.

**Figure 3:** Protein expression of autophagic markers following long-term supplementation with 4% pomegranates in APPsw/Tg 2576 The levels of autophagic markers, LC3 and bcl1, in the brains of mice fed 4% pomegranate diet for 15 months were determined using western blot analysis. Treatment I: Wild type (non-transgenic) control of the APPsw mice fed with regular diet; Treatment II: APPsw mice also fed with regular diet; and Treatment III: APPsw mice fed with 4% pomegranate fruit diet. **A.** The blot shown is representative tracings of an experiment done six times. **B.** Graphs are mean ± S.E brains from tissue obtained from six rodents for each treatment group. Each bar of the quantification graph represents the corresponding band for each age group. Significance ^*^p < 0.01 compared to wild-type mice fed with regular diet, ^#^*p* < 0.01 compared to APPsw transgenic mice fed with regular diet.

### The PI3K/Akt/mTOR signaling pathway is activated in APPsw/Tg 2576 treated with 4% pomegranates for 15 months

The activation of protein translation by the PI3K/Akt/mTOR signaling pathway is a key regulator of synaptic plasticity [52]. We assessed the effect of supplementation with 4% pomegranates on activation of the PI3K and mTOR by determining the phosphorylation levels of Akt and p70 S6 kinase (p70S6K) using immunoblotting. Our data shows that phosphorylation of Akt, mTOR and p70S6K were significantly increased in the brain of 4% pomegranate-treated APPsw/Tg 2576 mice compared to APPsw/Tg 2576 mice receiving a standard chow diet (*p* < 0.05) (Figure 4).

**Figure 4:** mTOR signaling pathway in brain homogenates detected by Western blot analysis The levels Akt, mTOR and p70S6K, and their phosphorylated forms in the brains of mice fed 4% pomegranate diet for 15 months. Treatment I: Wild type (non-transgenic) control of the APPsw mice fed with regular diet; Treatment II: APPsw mice also fed with regular diet; and Treatment III: APPsw mice fed with 4% pomegranate fruit diet. **A.** The blot shown is representative tracings of an experiment done six times. **B.** Graphs are mean ± S.E brains from tissue obtained from six rodents for each treatment group. Each bar of the quantification graph represents the corresponding band for each age group. Significance ^*^p < 0.01 compared to wild-type mice fed with regular diet, ^#^*p* < 0.01 compared to APPsw transgenic mice fed with regular diet.

### Treatment with 4% pomegranates lowered amyloidogenic processing of APP in APPsw/Tg 2576 after 15 months

We also investigated the effect of a 4% pomegranate dieton APP processing by Western blot (Figure 5). Increased APP anabolism may stimulate APP secretion. Therefore, we determined the effect of 4% pomegranate dieton full-length APP levels. We used a polyclonal carboxyl-terminal APP antibody that is specific to both Carboxyl-Terminal Fragment β (CTFβ) and Carboxyl-Terminal Fragment α (CTFα). No significant difference was observed on APP steady-state protein expression in the brains of APPsw/Tg 2576 fed standard chow diet, and APPsw/Tg 2576 mice administered a 4% pomegranate diet. This suggests that pomegranates and their constituents do not influence APP synthesis. BACE1 is responsible for the proteolytic cleavage of full length APP to form sAPPβ and CTFβ. We observed a significant increase in BACE1, sAPPβ, and CTFβ expression in the brains of APPsw/Tg 2576 compared to wild-type mice (*p*< 0.05). After treatment with a 4% pomegranate diet, the expression of BACE1, sAPPβ, and CTFβ in APPsw/Tg 2576 mice was significantly decreased after 15 months (*p* < 0.05).

The article "Consumption of pomegranates improves synaptic function in a transgenic mice model of Alzheimer's disease" was retracted in 2025. Reasons: duplicated images; original data or images not available; concerns about the images; concerns about the authorship.

CTFα is produced as a by-product of α-secretase cleavage, which is regulated by the metalloproteases, ADAM10 and ADAM17 [53-59]. The protein expression of CTFα was significantly increased by more than 2-fold in APPsw/Tg 2576 mice brains compared with wild-type controls (*p* < 0.05). However, no significant difference on the levels of CTFα, ADAM10 and ADAM17 was observed after pomegranatetreatment. This suggests that a pomegranate-rich diet has no effect on the modulation of the α-secretase pathway.

**Figure 5:** BACE1 and APP processing in brain homogenates detected by Western blot analysis The levels APP, BACE1, CTFα, CTFβ, sAPPβ, ADAM10 and ADAM17 in the brains of mice fed 4% pomegranate diet for 15 months. Treatment I: Wild type (non-transgenic) control of the APPsw mice fed with regular diet; Treatment II: APPsw mice also fed with regular diet; and Treatment III: APPsw mice fed with 4% pomegranate fruit diet. **A.** The blot shown is representative tracings of an experiment done six times. **B.**Graphs are mean ± S.E brains from tissue obtained from six rodents for each treatment group. Each bar of the quantification graph represents the corresponding band for each age group. Significance ^*^p < 0.01 compared to wild-type mice fed with regular diet, ^#^*p* < 0.01 compared to APPsw transgenic mice fed with regular diet.

## DISCUSSION

The present study demonstrated for the first time that pomegranate diet administered for 15 months enhanced synaptic plasticity by increasing the expression of synaptic proteins, including PSD-95, Munc18-1, SNAP25, synaptophysin, p-CaMKIIα/ CaMKIIα, and pCREB/CREB, inhibited neuroinflammation, promoted autophagy, activated PI3K-Akt-mTOR signaling pathway, and altered APP processing in APPsw/Tg 2576 mice.

The article "Consumption of pomegranates improves synaptic function in a transgenic mice model of Alzheimer's disease" was retracted in 2025. Reasons: duplicated images; original data or images not available; concerns about the images; concerns about the authorship.

The beneficial effects of fruits and vegetables in health and ageing have been well emphasized. However, few studies have demonstrated the neuroprotective effects of pomegranate consumption in preclinical and clinical trials for AD. Pomegranates have been shown to consist of numerous phytochemicals, with potent antioxidant and anti-inflammatory properties. Indeed, our qualitative analysis using high precision liquid chromatography (HPLC) has shown that pomegranate extracts contain active components in significant amounts of ellagitannin, such as punicalin and punicalagin, and flavonoids, such as kaempferol and quercetin derivatives (Data not shown). Apart from demonstrating potent antioxidant and anti-inflammatory properties, ellagic acid and punicalagin, are β-secretase inhibitors [60]. As well, recent studies have suggested that quercetin may exert its beneficial effects independent of its antioxidant properties. Quercetin can also modulate pathways associated with mitochondrial biogenesis, mitochondrial membrane potential, oxidative respiration and ATP anabolism, intra-mitochondrial redox status, and subsequently, mitochondria-induced apoptosis [61]. Taken together, the active phytochemicals present in pomegranate extracts possess beneficial effects on brain function and can mitigate different hallmarks of neurodegeneration.

We and others have previously shown that dietary pomegranate supplementation can attenuate chronic oxidative stress in APPsw/Tg 2576 mice, reduce acetylcholinesterase activity and plasma Aβ_1-40_ and Aβ_1-42_ levels, and ameliorate memory and anxiety-related behavioural deficits, and improve spatial learning ability *in vivo*, consistent with our findings [47-49]. Biological extracts derived from the pomegranate rind have been shown to inhibit BACE1 activity *in vitro*. Pomegranate consumption has also been shown to improve brain function in several neurodegenerative disease models [62]. For instance, pomegranates attenuated 1-methyl-4-phenyl-1,2,3,6-tetrahydropyridine-induced oxidative stress and apoptosis in neuronal cells [63]. Reduced brain damage was also observed in postnatal day 7 pups exposed maternally to hypoxic insult [45, 46, 64]. Improvements in motor behaviour have also been reported in mice exposed to cytotoxic levels of proton radiation following pomegranate consumption [65]. Ellagic acid possesses potent neuroprotective effects through its free radical scavenging properties, iron chelation, activation of different cell signaling pathways, and mitigation of mitochondrial dysfunction.

The article "Consumption of pomegranates improves synaptic function in a transgenic mice model of Alzheimer's disease" was retracted in 2025. Reasons: duplicated images; original data or images not available; concerns about the images; concerns about the authorship.

Synaptic loss represents another pathological hallmark in AD. It is well established that alterations in the expression of synaptic proteins precedes neuronal loss in AD [66-69]. Therefore, we analyzed the changes in protein expression of several important synaptic proteins associated with maintenance of normal plasticity. We found a significant reduction in the presynaptic marker synaptophysin and postsynaptic marker PSD-95 in APPsw/Tg 2576 mice after 15 months, and supplementation with a 4% pomegranate diet upregulated the expression of these proteins. Increased calcium influx through activated N-methyl-D-aspartate (NMDA) receptors induces autophosphorylation of Calcium/Calmodulin-Dependent Protein Kinase II (CaMKII), and enhances translocation of CaMKII to the post-synapse. This leads to the activation of Cyclic AMP-Response Element Binding Protein (CREB). This nuclear transcription factor is associated with the formation of long-term memory [70-75]. We found that the ratio of pCaMKIIα/CaMKIIα and pCREB/CREB declined in APPsw/Tg 2576 mice at 15 months compared to wild-type mice. However, supplementation with 4% pomegranates significantly improved the ratio of pCaMKIIα/CaMKIIα and pCREB/CREB declined in APPsw/Tg 2576 mice. Our data collectively suggests that a pomegranate-rich diet may attenuate deficits in memory and cognition through upregulation of signalling pathways associated with synaptic plasticity.

Inflammation has been shown to represent a double-edged sword in AD pathogenesis - it is deleterious to neurons, but is necessary to facilitate the clearance of neurotoxic Aβ deposits [76]. Upregulation of important inflammatory transcripts, *tnf-α*, *il-1β*, *iNOS*, *ccl2*, and *il-1* were observed in APPsw/Tg 2576 mice compared to wild-type mice. However, supplementation with 4% pomegranate diet reduced the expression of these proinflammatory gene transcripts. We also examined whether the anti-inflammatory effects of a pomegranate diet may be due to an autophagic-dependent effect. Our data shows that 4% pomegranate diet increased the protein expression of bcl1 and LC-3 type II. Bcl1 is an essential protein that enhances microglial phagocytosis, and autophagy is crucial for the catabolism of abnormal Aβ aggregates by activated microglial cells in the brain [77-80].

Another protein associated with synaptic plasticity is mTOR [81, 82]. Increased calcium influx through activated NMDA receptors can activate mTOR, thus promoting the anabolism of protein, including NR1, CaMKIIα, PSD-95, Arc, and protein kinase C isoform protein kinase M zeta, to stimulate synaptic plasticity [82-89]. Deregulation of mTOR signalling has been associated with cognitive and behavioural deficits [90-95]. Increased APP processing and the Aβ peptides can inhibit the PI3K-Akt-mTOR pathway, and reduced mTOR activity has been reported in both APPsw/Tg 2576 mice and human AD patients [96-116]. Likewise, we found that phosphorylation of mTOR was significantly decreased in 15 month old APPsw/Tg 2576 mice. These pathological changes were improved followingtreatment with 4% pomegranate diet. Therefore, another mechanism by which pomegranates may improve synaptic function may be through activation of the PI3K-Akt-mTOR pathway.

The article "Consumption of pomegranates improves synaptic function in a transgenic mice model of Alzheimer's disease" was retracted in 2025. Reasons: duplicated images; original data or images not available; concerns about the images; concerns about the authorship.

We also investigated whether a pomegranate diet can change the proteolytic processing of APP, by measuring the protein expression of BACE1. In line with previous studies, we found that BACE1 protein levels were significantly increased 15 month old APPsw/Tg 2576 mice compared to wild-type controls [62]. Treatment with 4% pomegranates significantly reduced BACE1 expression. Therefore, BACE1 inhibition may represent a valuable target for reducing Aβ levels in AD [117]. Additionally, the protein expression of sAPPβ and CTFβ, were also reduced 15 month old APPsw/Tg 2576 mice exposed to 4% pomegranate diet. These results provide additional support for the inhibitory effects of pomegranate consumption of BACE1 activity in AD.

The proteolytic cleavage of APP is initiated non-amyloidogenically by α-secretase. ADAM10 and ADAM17 are two main enzymes with α-secretase activity [118-120]. Although ADAM10 is necessary for APP α-secretase cleavage, ADAM17 may also be involved, although it is not crucial [121]. No significant difference in the expression of ADAM10 and ADAM17 were observed between 15 month old APPsw/Tg 2576 mice and wild-type mice. An increase in CTFα level observed in the APPsw/Tg 2576 mice compared to wild-type mice may be due to increased levels of APP, the α-secretase substrate, or α-secretase activity in APPsw/Tg 2576 mice. The expression of ADAM10, ADAM17, and CTFα, remained unchanged, following treatment with 4% pomegranates, suggesting that α-secretase activity is independent of pomegranate-mediated APP processing.

In conclusion, this study has demonstrated for the first time that long-term supplementation with a 4% pomegranate dietcan enhance synaptic plasticity in APPsw/Tg 2576 mice, leading to reduced cerebral Aβ levels, cleavage of CTFβ and sAPPβ, and BACE1 protein expression. Together with other mechanisms, such as inhibition of neuroinflammation, and increased autophagy, pomegranates may represent alternative treatment to lower AD pathology.

## MATERIALS AND METHODS

### Collection and preparation

Fresh pomegranate fruits were collected from Al-Jabal Al-Akdhar farms, Oman. Then, pomegranates were frozen (-40°C) for 5 days. After that, the samples were ground into a fine powder using a coffee grinder.

The article "Consumption of pomegranates improves synaptic function in a transgenic mice model of Alzheimer's disease" was retracted in 2025. Reasons: duplicated images; original data or images not available; concerns about the images; concerns about the authorship.

### Diet preparation for the animals

The ground pomegranates were sent to USA to prepare the diet for the mice. The diet was prepared by mixing the pomegranate (4%) with regular diet as per National Institutes of Health, USA protocol by Research Diet Inc, NJ, USA.

### Animals and treatment

Twelve transgenic female (APPsw/Tg 2576) and 6 wild-type control (non-transgenic) mice (Taconic form, NY, USA) were used. Animals were quarantined for 7 days after shipping and individually housed in plastic cages in an animal room, which was maintained at a temperature of 22±2°C, a relative humidity of 50±10%, and a 12-h light/dark automatic light cycle (light: 08:00-20:00 h). Tap water was offered *ad libitum* throughout the study. The study was approved by the Animal Care and Use Committee of the Sultan Qaboos University, Oman (SQU/AEC/2010-11/3).

All these animals are free from pathogens and viruses. Experimental period commenced from the age of 4 months. The animals were divided into three groups: Treatment I: Wild type (non-transgenic) control of the APPsw mice fed with regular diet; Treatment II: APPsw mice also fed with regular diet; and Treatment III: APPsw mice fed with 4% pomegranate fruit diet. These experimental and control mice were fed a 4% pomegranate or control diet for 15 months. All animal experiments in the present study were complied with the Animal Care and Use Committee of the Sultan Qaboos University, Oman.

### Tissue collection

The brains were carefully removed, and homogenization in 9 volumes (1:9 w/v) of cold saline, and centrifugation for supernatant collection. The samples of the brain were stored at −80°C until measurement.

### Reverse transcription and quantitative PCR for analysis of gene transcripts

For the gene expression studies RNA was extracted from treated human astrocytes and neurons using the RNeasy mini kits (Qiagen, Hilden, Germany). The cDNA was prepared using the SuperScript III First-Strand Synthesis System and random hexamers (Invitrogen Corporation). Q-PCR was carried out using the Mx3500P Real-Time PCR system (Stratagene, NSW, Australia) with the Taqman gene expression assays of mouse*tumour necrosis factor-α*tnf*-α)*, *interleukin 1-β*il*-1β)*,*inducible nitric oxide synthase* [122], chemokine (C-C motif) ligand 2 (ccl2), *interleukin 1-βil-10)*,*brain-derived neurotrophic factor (bdnf)*,*insulin-like growth factor (igf)-1*,*glyceraldehyde 3-phosphate dehydrogenase (gapdh)*(all from Life Technologies). at 4°C. The

### Western blotting

The brains of animals were dissected on ice and immediately processed. Briefly, hippocampal tissue were homogenized in RIPA buffer (50 mM, Tris-Cl, pH 7.5, 150 mM NaCl, 1% NP-40, 0.5% sodium deoxycholate, and 1% SDS), supplemented with a protease inhibitor cocktail (Sigma-Aldrich P8340) and phosphatase inhibitors (50 mM NaF, 1 mM Na_3_VO_4_ and 30 μM Na_4_P_2_0_7_), using a Potter homogenizer and then passed sequentially through different calibre syringes. Protein samples were centrifuged at 14000 rpm at 4°C twice for 15 min [26]. Protein concentration was determined using the BCA Protein Assay Kit (Pierce Biotechnology, Rockford, IL). 20 μg of hippocampal samples were resolved by 10% SDS-PAGE and transferred to a PVDF membrane. The reactions were followed by incubation with a primary antibody; then a secondary anti-goat peroxidase conjugated antibody (Pierce) was used and developed using an ECL kit (Western Lightning Plus ECL, PerkinElmer).

The article "Consumption of pomegranates improves synaptic function in a transgenic mice model of Alzheimer's disease" was retracted in 2025. Reasons: duplicated images; original data or images not available; concerns about the images; concerns about the authorship.

### Statistical analysis

Results are expressed as mean ± standard error. Data were analysed by one-way ANOVA, followed by Bonferroni's *post hoc* test. p≤0.05 was considered as statistically significant. Statistical analysis was performed using Prism software (GraphPad Software Inc).
